This article has been retracted.

# Effects of Four Types of Watermelon Frost Combination Medications for the Treatment of Oral Ulcers: A Network Meta-Analysis

**DOI:** 10.1155/2022/2712403

**Published:** 2022-03-12

**Authors:** Zhenhua Liu, Huiqin Dou

**Affiliations:** ^1^Department of Stomatology, Zhongguancun Hospital, Beijing 100080, China; ^2^Department of Oral Medicine, Qilu Hospital of Shandong University, Jinan 250012, China

## Abstract

**Objective:**

The aim of this study is to identify the effectiveness of the four different watermelon frost combination medications in the treatment of oral ulcers through network meta-analysis and rank them based on their performances.

**Methods:**

Five randomized controlled studies of four distinct types of a combination medication for the treatment of oral ulcers were observed in numerous databases, and a network meta-analysis was conducted to evaluate the odds ratio (OR) and sequence of the diverse treatments using Stata software (version 13.0). The underlined studies were categorized into two groups: the control group (watermelon frost alone) and the observation group (one of four watermelon frost combinations).

**Results:**

The study comprised of 598 cases and the findings indicated that the pooled OR and 95% CI of oral ulcers that improved relative to watermelon frost alone were 3.26 (1.28 to 8.30) for watermelon frost and Kangfuxin fluid, 8.74 (2.94 to 26.02) for watermelon frost and erythromycin, 6.53 (1.81 to 23.50) for watermelon frost and metronidazole, and 2.62 (0.63 to 10.95) for watermelon frost and cydiodine buccal tablets. The study showed the significant efficacy of watermelon frost combination medications. In terms of clinical efficacy, the combination of watermelon frost and erythromycin was the most promising concomitant medication. It had an 86.3 surface under cumulative ranking (SUCRA).

**Conclusion:**

All the studied watermelon frost combinations were effective against oral ulcers validating the use of watermelon frost for oral ulcers. The combination of watermelon frost and erythromycin is the most promising candidate among the four combinations for the treatment of oral ulcers.

## 1. Introduction

Oral ulcer is a common oral disease in clinics. It is a superficial ulcer that occurs on the oral mucosa. The ulcer is mainly round or oval. The common symptom is local oral pain. This disease has the highest incidence among oral mucosal diseases and has a certain periodicity and self-limitation [1]. At present, the etiological mechanism of the disease is not very clear, and may be closely related to heredity and infection. The disease will affect the patient's normal diet and even language function and cause great pain to the patient [2]. Improper treatment after the onset of the disease will significantly reduce the quality of life. If it is not treated timely and effectively, it is easy to involve diseases of the nervous, cardiovascular, digestive, and respiratory systems [3]. Therefore, the timely and effective clinical treatment of oral ulcer patients with scientific and reasonable treatment plans has very important clinical significance for enhancing the quality of life.

The meta-analysis, which is based on direct comparisons of well-planned randomized controlled trials, has been considered as the gold standard for determining the effectiveness of interventions [4]. In clinical practice, there is no evidence of direct comparative studies on the efficacy of many different interventions. The biggest advantage of network meta-analysis (NMA) is that distinct interventions for the treatment of the same disease can be indirectly compared and sorted according to the effect of a certain outcome index, and then, the optimal treatment plan can be selected [5, 6].

The current study aimed to identify the effectiveness of four types of watermelon frost combination medications for the treatment of oral ulcers using NMA and to rank them according to their performances. These four schemes are most widely used to treat oral ulcers. Watermelon frost spray is an anti-inflammatory Chinese patent medicine. This included combinations of watermelon frost with Kangfuxin fluid, erythromycin, metronidazole, and cydiodine buccal tablets. This study may provide critical guidance for therapeutic medication selection in the treatment of oral ulcers.

## 2. Methods

### 2.1. Search Strategy

The databases conducted for this research included EMBASE, PubMed, Web of Science, China Science and Technology Journal, SciFinder, Sino Med, Wan fang, China National Knowledge Index, China Academic Journal Network Publishing, Chinese Science Citation, Cochrane Library, China Biomedical Medicine, Chongqing VIP Network, and BIOSIS Previews. Each database has its own set of search algorithms, which include variations on the search keywords, wildcard symbols, and Boolean operators that combine words. The searching date is from the establishment of the database to February 17, 2021. The searched words are “watermelon frost,” “combination therapy,” “Kangfuxin fluid,” “erythromycin,” “metronidazole,” “cydiodine buccal tablets,” “oral ulcer,” “mouth ulcer,” “aphthous,” “randomized controlled trials,” “efficacy,” and “drug therapy.”

### 2.2. Inclusion and Exclusion Criteria

The following were the inclusion criteria: (1) randomly controlled trials, (2) subjects with oral ulcers who met the requirement of diagnosis of oral ulcers [7]: the integrity of the oral mucosal epithelium is continuously damaged or destroyed, and the surface layer is necrotic and sloughed to form a depression [8], (3) patients aged 18 years and above, (4) the results of the effective number of cases of both the observation group and the control group are provided, (5) absence of seriously malignant ulcers, and (6) studies in which watermelon frost alone was used as the control group and watermelon frost combinations were utilized to treat oral ulcers as the observation group.

The following were the exclusion criteria: (1) subjects with tuberculous ulcer, traumatic ulcer, oral mucosa herpes simplex, or mental illness, (2) individuals with serious tumor, heart, kidney, lung, or liver damage, as well as those with autoimmune illnesses (3) studies that are entirely descriptive and do not include a control group, (4) types of studies that were theoretical reviews, discussions of case reports, and summaries of experience, and (5) studies in which incomplete data are provided.

### 2.3. Efficacy Evaluation Criteria

The efficacy was assessed using the integral value of clinical signs and indicators pre- and post-treatment: (1) healed: the ulcer surface was completely healed, and the clinical symptoms and signs disappeared; (2) markedly effective: the ulcer surface was obviously healed. Moreover, the clinical symptoms and indications had improved noticeably; (3) effective: the ulcer surface was partially healed, and the clinical symptoms and signs were partially improved; (4) ineffective: the ulcer surface was not healed or even enlarged, and the clinical symptoms and signs remained unchanged or even worsened. The total effective cases were the sum of effective, markedly effective, and healed cases.

### 2.4. Data Extraction and Quality Evaluation

Two reviewers read the literature independently and searched all titles and abstracts of potentially eligible trials based on the inclusion and exclusion criteria, and then they extracted all relevant information including numerical results, sample size (control and observation) in each arm, characteristics of participants and interventions, outcomes reported and collected, and quality indicators of publications in each included study. The information extracted was cross-checked and disagreements were transferred to a third reviewer. The quality of the publications in this study was assessed using the Jadad quality scoring system.

### 2.5. Statistical Evaluations

The network meta-analysis was used by using Stata software 13.0 version to construct the network commands network package was used to construct evidence contribution, forest plot, funnel, and ranking plots. The value of the SUCRA curve was used to rank the efficacy of the interventions. SUCRA values were shown in percentages. The greater the SUCRA value, the better the intervention. The selected indicators were count data, while ORs were used as the concomitant effect, and CIs were set at 95%. The probability value of *P* < 0.05 was regarded as statistically considerable.

### 2.6. Ethical Approval and Consent to Participate

Each study was based on a previously published research study. As a result, there was no need for ethical approval or patient consent.

## 3. Results

### 3.1. Characteristics of Included Studies

This study eventually identified 5 eligible publications published between 2016 and 2020. A total of 598 cases including 299 observation cases and 299 control cases were included. The basic classification of included papers is shown in Table 1.

### 3.2. Network Meta-Analysis

#### 3.2.1. Network Plot of Four Types of Integrated Chinese and Western Medicines

Of the 5 studies, the combination of watermelon frost with Kangfuxin fluid was the most common one, while watermelon frost with erythromycin, metronidazole, and cydiodine buccal tablets were the least, all were one.  Figure 1 showed that the watermelon frost alone group had the largest number of participants, while watermelon frost with cydiodine buccal tablets had the least number of subjects.

#### 3.2.2. Evidence Contribution Plot

The direct comparison of watermelon frost alone and the combination of watermelon frost + Kangfuxin fluid had a 100% impact on the combined results. The direct comparison between watermelon frost alone and watermelon frost + Kangfuxin fluid had a 50% effect on the indirect comparison between watermelon frost + Kangfuxin fluid and watermelon frost + erythromycin. The direct comparison of watermelon frost alone and watermelon frost + Kangfuxin fluid had a 16.7% effect on the results of the meta-analysis (Figure 2).

#### 3.2.3. Forest Plot

The pooled OR and 95% CI of oral ulcers improvement compared with watermelon frost alone was 3.26 (1.28 to 8.30) for watermelon frost + Kangfuxin fluid, 8.74 (2.94 to 26.02) for watermelon frost + erythromycin, 6.53 (1.81 to 23.50) for watermelon frost + metronidazole, and 2.62 (0.63 to 10.95) for watermelon frost + cydiodine buccal tablets, considerably, which shows considerable variations in efficacy. For the comparison between watermelon frost combinations, no considerable variations were observed. The OR for the network estimates along with 95% CI is shown in Figure 3.

#### 3.2.4. Publication Bias

In terms of publishing bias, all of the study's outcomes were nearly symmetrical (Figure 4), implying that there was no publication bias.

### 3.3. Ranking Plot

Table 2 and Figure 5 illustrate the distribution of probability for each treatment that was ranked for its efficacy in treating oral ulcers based on SUCRA values. The following was the order of SUCRA values for various watermelon frost combinations: watermelon frost + erythromycin (86.3), watermelon frost + metronidazole (75.0), watermelon frost + Kangfuxin fluid (46.8), and watermelon frost + cydiodine buccal tablets (39.4). As a result, the combination of watermelon frost and erythromycin had the best chance of being the most effective intervention in terms of clinical efficacy.

## 4. Discussions

Traditional meta-analysis is a direct head-to-head comparison of the treatment or safety of two treatment methods [9]. However, in practice, there are often many drugs to treat the same disease. Decision-makers, doctors, and patients need to be able to choose the best treatment method among a variety of treatment measures or programs [2]. Network meta-analysis is an extension of traditional meta-analysis and can be used to compare any number of treatments at the same time. Even if the two treatments to be compared have never been directly compared, this analysis method can still summarize the data of random clinical trials of different treatments, and then estimate the point and confidence interval for a given treatment endpoint [1,10].

In this research, four types of combined medicines with watermelon frost for treatment of oral ulcers were analyzed and pairwise comparison was performed to draw a network diagram, which showed a more intuitive result. The combinations of watermelon frost with Kangfuxin fluid, erythromycin, metronidazole, and cydiodine buccal tablets were more effective relative to watermelon frost alone in the treatment of oral ulcers. Watermelon frost combined with erythromycin had the greatest SUCRA value and was most likely to be the optimal treatment option.

The oral ulcer is a common oral mucosal disease in the hospital's oral departments [11]. It has the characteristics of recurring attacks, which make the patient feel very painful and has a serious impact on the daily life, study, and work of the patient [12]. The causes of oral ulcers mainly include two points: the first is that the oral cavity is infected by bacteria or viruses, which leads to oral mucosal erosion and ulcers; the second is that the patient's immune response causes oral mucosal ulcers [13, 14].

At present, the methods of clinical treatment of oral ulcers include traditional Chinese medicine treatment, western medicine treatment, and integrated traditional Chinese and western medicine treatment [15]. Clinically, watermelon frost sprays are often used to treat patients. The watermelon frost spray is made from traditional Chinese medicine, which contains 14 kinds of Chinese medicine including cork, sophora tonkinensis, scutellaria, coptis, menthol, fritillaria thunbergii, borneol, and borax. Borax in the composition has detoxification and antiseptic effects; fritillaria thunbergii can reduce swelling and anti-inflammatory; menthol and borneol have the effects of reducing swelling and pain, detoxification, and purging fire; the three herbs of phellodendron chinense, coptis, and scutellaria can be anti-inflammatory in action; sophora tonkinensis can also reduce swelling, relieve pain, and detoxify [16]. A variety of Chinese medicinal materials are mixed, so watermelon frost has a good effect of clearing heat and detoxification, reducing swelling and pain, clearing the throat and throat, promoting mucosal regeneration, and has a good therapeutic effect on oral ulcers.

However, a single drug cannot achieve the ideal therapeutic effect for the treatment of oral ulcers. In clinical practice, a combination of drugs is often used to improve the therapeutic effect and quickly relieve the pain of patients. Kangfuxin liquid belongs to a kind of traditional Chinese medicine biological preparation, which contains abundant mucosine, peptides, polyols, and other biologically active substances [17]. Metronidazole can affect the DNA metabolism process of bacteria, promote cell death, and has a good antibacterial effect. Cydiodine buccal tablets are mainly active iodine, which is quickly released after reacting with saliva, halogenating the protein of the bacteria, thereby achieving the effect of eliminating microorganisms [18]. This article found that the combination of watermelon frost and erythromycin is the best treatment option for oral ulcers. The combination regimen is putting erythromycin and watermelon frost together in a mortar, pounding it into a fine powder, then putting it in a powder spray bottle, shaking it evenly, and spraying it on the surface of the ulcer. Erythromycin is a macrolide antibiotic extracted from the culture medium of Streptomyces erythreus [19]. From the analysis of pharmacological effects, it is the use of erythromycin to bind to the 50S subunit of the bacterial ribosome, inhibit peptide acyltransferase, and then affect the translocation of ribonucleosome. The process hinders the growth of the peptide chain and ultimately inhibits the synthesis of bacterial protein to control secondary infections [20].

### 4.1. Limitations of the Study

Although this study has the potential to be highly useful in the clinical treatment of oral ulcers, it has certain limitations. The side effects of the four concomitant drugs with watermelon frost were not reported in studies. Therefore, their results were not analyzed. The research only looks at Chinese studies and there is no quantitative analysis of immune system cytokines. Therefore, high-quality randomized controlled trials are needed in the future to evaluate the efficacy of combining medicines and watermelon frost in oral ulcers.

## 5. Conclusion

The oral ulcer is a common oral disease-causing superficial round or oval ulcer that occurs on the oral mucosa with a common symptom of local oral pain. Watermelon frost has traditionally been used for the treatment of oral ulcers. This study was designed to identify the effectiveness of four types of watermelon frost combination medications for the treatment of oral ulcers using NMA and to rank them according to their performances. These four schemes are most widely used to treat oral ulcers. Watermelon frost spray is an anti-inflammatory Chinese patent medicine. This included combinations of watermelon frost with Kangfuxin fluid, erythromycin, metronidazole, and cydiodine buccal tablets. Five randomized controlled studies of four distinct types of a combination medication for the treatment of oral ulcers were evaluated using network meta-analysis (NMA). The underlined studies were categorized into two groups: the control group (watermelon frost alone) and the observation group (one of four watermelon frost combinations). The study showed the significant efficacy of watermelon frost combination medications. In terms of clinical efficacy, the combination of watermelon frost and erythromycin was the most promising concomitant medication with 86.3 surfaces under cumulative ranking (SUCRA). This study may provide critical guidance for therapeutic medication selection in the treatment of oral ulcers. A combination of watermelon frost with erythromycin is the most promising candidate among four combinations for the treatment of oral ulcers.

## Figures and Tables

**Figure 1:** Network plot of different interventions for treatment of acute cerebral infarction. The size of the point in the network graph is proportional to the number of subjects, while the thickness of the line is proportional to the number of studies. A, watermelon frost; B, watermelon frost + Kangfuxin fluid; C, watermelon frost + erythromycin; D, watermelon frost + metronidazole; E, watermelon frost + cydiodine buccal tablets.

**Figure 2:** Evidence contribution plot. The matrix showed the effect of comparing the results of different control measures directly against the results of their network meta-analysis. A, watermelon frost; B, watermelon frost + Kangfuxin fluid; C, watermelon frost + erythromycin; D, watermelon frost + metronidazole; E, watermelon frost + cydiodine buccal tablets.

**Figure 3:** Network estimates of mean OR, their 95% Cis, and prediction intervals (red extensions). A, watermelon frost; B, watermelon frost + Kangfuxin fluid; C, watermelon frost + erythromycin; D, watermelon frost + metronidazole; E, watermelon frost + cydiodine buccal tablets.

**Figure 4:** Funnel plot for publication bias in selected studies.

**Figure 5:** SUCRA for the cumulative probabilities. Notes: A, watermelon frost; B, watermelon frost + Kangfuxin fluid; C, watermelon frost + erythromycin; D, watermelon frost + metronidazole; E, watermelon frost + cydiodine buccal tablets.

**Table 1:** Classification of included studies.

Author	Comparison	Year	Area	Dose		Observation group		Control group		Duration (days)	Jadad quality score
				A	Combined medication	Total effective cases	Total cases	Total effective cases	Total cases		
Chen HZ	B vs A	2016	China	4 time/day	20 ml/day	37	40	32	40	7	3
You Ying	B vs A	2018	China	4 time/day	12–20 ml/day	36	40	29	40	7	4
Xu HF	C vs A	2013	China	4 time/day	4 time/day	101	105	78	105	7–14	3
Li XY	D vs A	2020	China	3 time/day	3 time/day	71	74	58	74	14	3
Shan HZ	E vs A	2014	China	6time/day	7.5 mg/day	37	40	33	40	7	3

A, watermelon frost; B, watermelon frost + Kangfuxin fluid; C, watermelon frost + erythromycin; D, watermelon frost + metronidazole; E, watermelon frost + cydiodine buccal tablets.

**Table 2:** SUCRA rankings of acute cerebral infarction treatments.

Treatment	SUCRA	PrBest	Mean rank
Watermelon frost	2.5	0.0	4.9
Watermelon frost + erythromycin	86.3	58.2	1.5
Watermelon frost + metronidazole	75.0	33.6	2.0
Watermelon frost + Kangfuxin fluid	46.8	3.1	3.1
Watermelon frost + cydiodine buccal tablets	39.4	5.1	3.4

Notes: SUCRA: surface under the cumulative ranking.

## Data Availability

The data used to support the findings of this study are available from the corresponding author upon request..
